# Association between the *TIMD4-HAVCR1* variants and serum lipid levels, coronary heart disease and ischemic stroke risk and atorvastatin lipid-lowering efficacy

**DOI:** 10.1042/BSR20171058

**Published:** 2018-01-19

**Authors:** Qing-Hui Zhang, Rui-Xing Yin, Wu-Xian Chen, Xiao-Li Cao, Yu-Ming Chen

**Affiliations:** 1 Department of Cardiology, Institute of Cardiovascular Diseases, The First Affiliated Hospital, Guangxi Medical University, Nanning 530021, Guangxi, China; 2 Department of Neurology, The First Affiliated Hospital, Guangxi Medical University, Nanning 530021, Guangxi, China

**Keywords:** coronary heart disease, genetic variants, hepatitis A virus cellular receptor 1, ischemic stroke, lipids, T-cell immunoglobulin domain and mucin domain 4

## Abstract

Little is known about the association of the *TIMD4* (T-cell immunoglobulin and mucin domain 4 gene)-*HAVCR1* (hepatitis A virus cellular receptor 1) variants and lipid metabolism, the risk of coronary heart disease (CHD) and ischemic stroke (IS). The present study aimed to determine the *TIMD4-HAVCR1* variants, their haplotypes and gene–environment interactions on serum lipid levels, the risk of CHD and IS, and the lipid-lowering efficacy of atorvastatin in a southern Chinese Han population. Genotypes of three variants in 622 controls, 579 CHD, and 546 IS patients were determined by the Snapshot technology. Atorvastatin calcium tablet (20 mg/day) was given in 724 hyperlipidemic patients for 8 weeks after genotyping. The rs12522248 genotypic and allelic frequencies were different between controls and patients, and were associated with the risk of CHD and IS. The rs1501908G-rs12522248T-rs2036402T haplotype was associated with an increased risk of CHD; the G-C-T haplotype was associated with lower risk of CHD; and the C-C-C haplotype was associated with an increased risk of IS. Variants and their haplotypes in controls were associated with triglyceride (rs1501908), low-density lipoprotein cholesterol (LDL-C, rs1501908, G-T-T), high-density lipoprotein cholesterol (HDL-C, rs12522248, C-C-C) and the ratio of total cholesterol (TC) to HDL-C (C-C-C). Interactions of rs1501908- and rs2036402-alcohol (HDL-C); rs1501908- and rs12522248-high body mass index (hBMI, ≥24 kg/m^2^; TC); and *TIMD4-HAVCR1* variants-atorvastatin on several lipid parameters were detected. Interactions of rs12522248TC/CC-hBMI, G-T-T-, and C-C-C-smoking on the risk of CHD; and C-C-C-smoking, C-C-C-, and G-C-T-hBMI on the risk of IS were also observed. These findings suggest that the *TIMD4-HAVCR1* variants may be the genetic risk factors for CHD and IS.

## Introduction

Coronary heart disease (CHD) and ischemic stroke (IS) remain the leading causes of morbidity and mortality globally [1,2]. The pathological basis of both diseases is atherosclerosis [3], which is a chronic process characterized by the combination of lipid accumulation and inflammatory immune processes in the arterial wall [4]. Atherogenic dislipidemia including elevated serum levels of total cholesterol (TC), triglyceride (TG), low-density lipoprotein cholesterol (LDL-C) and apolipoprotein (Apo) B, and low levels of high-density lipoprotein cholesterol (HDL-C). ApoA1 is a serious risk factor for atherosclerotic vascular diseases [5–10]. Both blood lipid disorder and atherosclerotic disease are multifactorial and complicated diseases caused by genetic factors [11,12], environmental factors [13–16], and their interactions [17–19]. Family history and twin studies showed that almost 40–70% of the interindividual variation in plasma lipid phenotypes [20,21] and 30–60% of the incidence of CHD and IS [22] can be explained by genetic factors, suggesting a considerable genetic contribution. Therefore, single nucleotide polymorphisms (SNPs) in the lipid-related genes [12,23,24] may have some associations with serum lipid levels, and the risk of CHD and IS.

The T-cell immunoglobulin and mucin domain 4 gene (*TIMD4*) and the hepatitis A virus cellular receptor 1 gene (*HAVCR1*; also known as *TIMD1*), the associated interval spanned two genes [24], are located on chromosome 5q23 and are members of the T-cell immunoglobulin domain and mucin domain gene family that plays a critical role in regulating immune responses. *TIMD4* is exclusively expressed on antigen-presenting cells, where it mediates phagocytosis of apoptotic cells and plays an important role in maintaining tolerance [25]. In contrast, *HAVCR1*, an important susceptibility gene for asthma and allergy, is preferentially expressed on T-helper 2 (Th2) cells and functions as a potent costimulatory molecule for T-cell activation [25]. Blockade of *TIMD4* and *HAVCR1* enhanced the risk of atherosclerosis in LDL receptor-deficient mice [26]. Genome-wide association study (GWAS) and other studies performed in different populations have reported that the *TIMD4-HAVCR1* variants were associated with serum lipid traits, but the association was inconsistent [24,27–29]. In addition, little is known about the association of the *TIMD4-HAVCR1* SNPs and the risk of CHD and IS. Therefore, the purpose of the present study was to detect the association of three SNPs (rs1501908, rs12522248, and rs2036402) in or near *TIMD4-HAVCR1*, their haplotypes and G × E interactions on serum lipid traits, the risk of CHD and IS, and the lipid-lowering efficacy of atorvastatin in a southern Chinese Han population.

## Materials and methods

### Study patients

A total of 1125 unrelated patients with CHD (*n*=579) and IS (*n*=546) were recruited from hospitalized patients in the First Affiliated Hospital, Guangxi Medical University. The diagnosis of CHD was based on typical ischemic discomfort plus one or more of electrocardiographic change (ST-segment depression or elevation of ≥0.5 mm, T-wave inversion of ≥3 mm in ≥3 leads or left bundle branch block), as well as increase in the cardiac markers, including creatinine kinase-MB and troponin T. Coronary angiography was performed in patients with CHD. The coronary angiograms were reviewed by two independent angiographers who were blinded to the results of the genotypes. For a vessel to be scored, stenosis ≥50% had to be noted in an epicardial coronary vessel of interest or in one of its major branches. In the event of discordance of the number of vessels scored between the two reviewers, angiograms were scored by a third independent reviewer. The selected CHD patients were subject to significant coronary stenosis (≥50%) in at least either one of the three main coronary arteries or their major branches (branch diameter ≥2 mm). Additionally, angiographic severity of disease was classified according to the number of coronary vessels with significant stenosis (luminal narrowing ≥50%) as one-, two- or three-vessel disease in the three major coronary arteries [30,31]. The diagnosis and classification of IS was ascertained in accordance with the TOAST (Trial of Org 10172 in Acute Stroke Treatment) criteria [32] after strict neurological examination, computed tomography, or MRI. The selected IS patients in the study included individuals who were eligible for one of the two subtypes of TOAST criteria: large-artery atherosclerosis and small-vessel occlusion. Individuals with a history of hematologic or brain MRI revealing cerebral hemorrhage, cardioembolic stroke, or unspecified stroke, neoplastic or intracranial space-occupying lesion, infection and other types of intracranial lesions, renal, liver, thyroid, autoimmune diseases, and type I diabetes were excluded. The selected IS patients who had a past history of CHD or IS were excluded from the study.

### Control subjects

A total of 622 control subjects matched by age, gender, and ethnic group were randomly selected from the healthy adults who underwent periodical medical check-up at the Physical Examination Center of the First Affiliated Hospital, Guangxi Medical University during the same period when CHD and IS patients were recruited. The controls were free of CHD and IS by questionnaires, history-taking, and clinical examination. The examination comprised physical examination, blood sampling, electrocardiography, chest X-ray, and Doppler echocardiography. All enrolled individuals were Han Chinese from Guangxi, the People’s Republic of China. Information on demography, socioeconomic status, medical history, and lifestyle factors was collected by trained research staff with standardized questionnaires for all participants. The reported investigations were in accordance with the principles of the Declaration of Helsinki. All procedures of the investigation were carried out following the rules of the Declaration of Helsinki of 1975 (http://www.wma.net/en/30publications/10policies/b3/), revised in 2008. The study design was approved by the Ethics Committee of the First Affiliated Hospital, Guangxi Medical University (number: Lunshen-2011-KY-Guoji-001; 7 March 2011). All procedures were performed in accordance with ethical standards. Informed consent was obtained from all participants.

### Atorvastatin treatment

A total of 724 hyperlipidemic patients (TC >5.17 mmol/l, and/or TG >1.70 mmol/l; 253 from control, 248 from CHD and 223 from IS) were treated with atorvastatin calcium tablet (Lipitor, Pfizer Wuxi Pharmaceutical Co., Ltd.) 20 mg per day for 8 weeks after the genotype determination. Blood samples were collected after 8 weeks of treatment again. Clinical biochemistry analyses for serum lipid profiles were performed.

### Biochemical measurements

Venous blood samples were obtained from all subjects after at least 12 h of fasting. The levels of serum TC, TG, HDL-C, and LDL-C in samples were determined by enzymatic methods with commercially available kits, Tcho-1, TG-LH (Randox Laboratories Ltd., Ardmore, Diamond Road, Crumlin Co., Antrim BT29 4QY, U.K., ), Cholestest N HDL and Cholestest LDL (Daiichi Pure Chemicals Co., Ltd., Tokyo, Japan), respectively. Serum ApoA1 and ApoB levels were detected by the immunoturbidimetric immunoassay (Randox Laboratories Ltd.). All determinations were performed with an autoanalyzer (Type 7170A; Hitachi Ltd., Tokyo, Japan) in the Clinical Science Experiment Center of the First Affiliated Hospital, Guangxi Medical University [33–36].

### Diagnostic criteria

The diagnosis of type II diabetes mellitus was based on the WHO diagnostic criteria for diabetes: (i) fasting plasma glucose (FPG) ≥7.0 mmol/l; (ii) Two-hour postprandial glucose ≥11.1 mmol/l; or (iii) self-reported diagnosis of diabetes or use of antidiabetic medications [37,38]. The individuals with TC >5.17 mmol/l, and/or TG >1.70 mmol/l were defined as hyperlipidemic [39,40]. Hypertension was defined according to the criteria outlined by the 1999 World Health Organization-International Society of Hypertension Guidelines for the management of hypertension [41,42]. Hypertension was defined as a systolic blood pressure of 140 mmHg or greater, and/or a diastolic blood pressure of 90 mmHg or higher, or the use of antihypertensive drugs. Normal weight, overweight, and obesity were defined as a body mass index (BMI) <24, 24–28, and >28 kg/m^2^, respectively [43,44].

### SNP selection and genotyping

The SNPs were selected on the basis of the following assumptions: (i) selected SNPs were established by Haploview (Broad Institute of MIT and Harvard, U.S.A., version 4.2); (ii) Information of the SNPs was obtained from NCBI dbSNP Build 132 (http://www.Ncbi.nlm.nih.gov/SNP/); (iii) SNPs were restricted to minor allele frequency (MAF) >1%. (iv) SNPs might be associated with the plasma lipid levels in recent GWASs [24,28]. Genomic DNA was extracted from leukocytes of venous blood using the phenol-chloroform method, and then sent to the Center for Human Genetics Research, Shanghai Genesky Bio-Tech Co. Ltd. Genotyping of the SNPs was performed by the Snapshot technology platform [33–36]. The restriction enzymes for the SNPs were SAP (Promega) and Exonuclease I (Epicentre), respectively. The sense and antisense primers were: rs1501908F: 5′-TTCTGTTAGGCCCTGAGAATAAAGACA-3′, rs1501908R: 5′-TGCCATTTACCAGA AAGAAAGTATTGGTA-3′; rs12522248F: 5′-AGGCCTTTGGGCTTCCAAACA-3′, rs12522248R: 5′-G TTCGAACGAGCACCACTGTTC-3′; rs2036402F: 5′-TGGGGAGAC AAA GGGAA GTCGT-3′, and rs2036402R: 5′-TGGGTGTCATCATTGCCAAAAG-3′.

### Statistical analyses

The statistical analyses were carried out using the statistical software package SPSS 17.0 (SPSS, Inc., Chicago, Illinois). Quantitative variables were expressed as mean ± S.D. (serum TG levels were presented as medians and interquartile ranges). Qualitative variables were expressed as percentages. Allele frequency was determined via direct counting, and the standard goodness-of-fit test was used to test the Hardy–Weinberg equilibrium (HWE). A chi-square analysis was used to evaluate the difference in genotype distribution and sex ratio between the groups. The general characteristics between patient and control groups were tested by the Student’s unpaired *t* test. The association of genotypes and serum lipid parameters was tested by analysis of covariance (ANCOVA) for TC, HDL-C, LDL-C, TC/HDL-C, ApoA1, ApoB, and ApoA1/ApoB and Kruskal–Wallis test for TG. Any variants associated with the serum lipid parameter at a value of *P*<0.017 (corresponding to *P*<0.05 after adjusting for three independent tests by the Bonferroni correction) were considered statistically significant. Unconditional logistic regression was used to assess the correlation between the risk of CHD and IS and genotypes. Age, gender, BMI, smoking, and alcohol consumption were adjusted for the statistical analysis. Odds ratio (OR) and 95% confidence interval (95% CI) were calculated using unconditional logistic regression. The interactions of three SNPs with alcohol consumption, cigarette smoking, BMI ≥24 kg/m^2^, age, and sex on serum lipid levels and the risk of CHD and IS were detected by using a factorial regression analysis [45–49]. After controlling for potential confounders, a *P*_I_≤0.003 was considered statistically significant after Bonferroni correction (according to three SNPs and five interactive factors). Pairwise linkage disequilibria and haplotype frequencies amongst the SNPs were analyzed using Haploview (Broad Institute of MIT and Harvard, U.S.A., version 4.2).

## Results

### General characteristics

The general characteristics of the patients and healthy controls are summarized in Table 1. The values of BMI, systolic blood pressure, pulse pressure, TG, and the ratio of TC to HDL-C were higher, but diastolic blood pressure, TC, HDL-C, ApoA1, the percentage of alcohol consumption, and the ratio of ApoA1 to ApoB were lower in CHD patients than in controls (*P*<0.05–0.001). The values of BMI, systolic blood pressure, diastolic blood pressure, pulse pressure, TG, and the ratio of TC to HDL-C were higher, whereas those of TC, HDL-C, ApoA1, the percentage of alcohol consumption, and the ratio of ApoA1 to ApoB were lower in IS patients than in controls (*P*<0.05–0.001).

**Table 1:** Comparison of general characteristics and serum lipid levels between controls and patients

Parameter	Control	CHD	IS	*P*_CHD_	*P*_IS_
Number	622	579	546	-	-
Male/female	446/176	431/148	394/152	0.286	0.862
Age, years	61.68 ± 11.99	62.23 ± 10.56	62.87 ± 12.34	0.403	0.097
BMI, kg/m^2^	22.64 ± 3.20	23.89 ± 3.22	23.39 ± 3.49	<0.001	<0.001
Systolic blood pressure, mmHg	127.39 ± 19.77	133.05 ± 23.29	147.63 ± 22.16	<0.001	<0.001
Diastolic blood pressure, mmHg	81.28 ± 13.08	79.15 ± 14.20	83.73 ± 12.97	0.007	0.001
Pulse pressure, mmHg	46.11 ± 18.27	53.90 ± 17.50	63.89 ± 17.92	<0.001	<0.001
Cigarette smoking, *n* (%)	248 (39.9)	250 (43.2)	227 (41.6)	0.245	0.554
Alcohol consumption, *n* (%)	267 (42.9)	134 (23.1)	152 (27.8)	<0.001	<0.001
TC, mmol/l	4.99 ± 1.06	4.53 ± 1.19	4.52 ± 1.14	<0.001	<0.001
TG, mmol/l	1.00 (0.71)	1.36 (0.94)	1.36 (0.92)	<0.001	<0.001
HDL-C, mmol/l	1.90 ± 0.50	1.14 ± 0.033	1.23 ± 0.40	<0.001	<0.001
LDL-C, mmol/l	2.77 ± 0.78	2.71 ± 1.00	2.70 ± 0.89	0.272	0.163
TC/HDL-C	2.77 ± 1.26	4.22 ± 1.84	3.96 ± 1.44	<0.001	<0.001
ApoA1, g/l	1.41 ± 0.27	1.04 ± 0.52	1.03 ± 0.22	<0.001	<0.001
ApoB, g/l	0.90 ± 0.21	0.91 ± 0.27	0.89 ± 0.24	0.713	0.455
ApoA1/ApoB	1.65 ± 0.52	1.38 ± 2.48	1.25 ± 0.58	0.009	<0.001
Type II diabetes mellitus, *n* (%)	25 (4.0)	95 (16.3)	124 (22.3)	<0.001	<0.001
Hypertension, *n* (%)	180 (28.7)	298 (51.0)	272 (49.0)	<0.001	<0.001

The value of TG was presented as median (interquartile range), the difference between CHD/IS patients and controls was determined by the Wilcoxon–Mann–Whitney test. Abbreviations: *P*_CHD_, CHD compared with controls; *P*_IS_, IS compared with controls.

### Genotypic and allelic frequencies

The genotypic and allelic frequencies of the three *TIMD4-HAVCR1* SNPs are presented in Table 2. The genotype distribution of the three SNPs was concordant with the HWE in patients and controls (*P*>0.05 for all). The genotypic and allelic frequencies of the rs12522248 SNP were different between controls and patients (CHD and IS, *P*<0.05 for all). There was no difference in the genotypic and allelic frequencies of the rs1501908 and rs2036402 SNPs between CHD or IS patients and controls (*P*>0.05 for each). Significant linkage disequilibrium (LD) was noted between the rs1501908 and rs2036402 SNPs; and between rs12522248 and rs2036402 SNPs in controls and patients (*D′*>0.8).

**Table 2:** Genotypic and allelic frequencies of three SNPs in controls and patients (*n* (%))

SNP	Control	CHD	IS	*P*_CHD_	*P*_IS_
	*n*=622	*n*=579	*n*=546		
**rs1501908**					
CC	307 (49.4)	286 (49.4)	296 (54.2)		
CG	264 (42.4)	235 (40.6)	204 (37.4)		
GG	51 (8.2)	58 (10.0)	46 (8.4)	0.512	0.200
C	878 (70.6)	807 (69.7)	796 (72.9)		
G	366 (29.4)	351 (30.3)	296 (27.1)	0.634	0.215
*P*_HWE_	0.583	0.345	0.203		
**rs12522248**					
TT	472 (75.9)	384 (66.3)	376 (68.9)		
TC	137 (22.0)	170 (29.4)	149 (27.3)		
CC	13 (2.1)	25 (4.3)	21 (3.8)	0.001	0.015
T	1081 (86.9)	938 (81.0)	901 (82.5)		
C	163 (13.1)	220 (19.0)	191 (17.5)	<0.001	0.003
*P*_HWE_	0.414	0.268	0.203		
**rs2036402**					
TT	496 (79.7)	459 (79.3)	430 (78.8)		
TC	119 (19.1)	117 (20.2)	105 (19.2)		
CC	7 (1.1)	3 (0.5)	11 (2.0)	0.469	0.466
T	1111 (90.8)	1035 (89.4)	965 (88.4)		
C	133 (9.2)	123 (10.6)	127 (11.6)	0.965	0.472
*P*_HWE_	0.963	0.122	0.132		

Abbreviations: *P*_CHD_, CHD compared with controls; *P*_IS_, IS compared with controls.

### *TIMD4-HAVCR1* genotypes and the risk of CHD and IS

As shown in Figure 1, the genotypes of the rs12522248, but not the other two SNPs, were associated with the risk of CHD after the Bonferroni correction (a value of *P*<0.017 was considered statistically significant) in different genetic models: dominant: CT/CC compared with TT (OR =1.43, 95% CI =1.10–1.88, *P*=0.0084) and log-additive model: C compared with T (OR =1.39, 95% CI =1.10–1.75, *P*=0.0052). The genotypes of the rs12522248 SNP were also associated with the risk of IS in different genetic models: dominant model: CT/CC compared with TT (OR =1.43, 95% CI =1.10–1.86, *P*=0.0082) and log-additive model: C compared with T (OR =1.39, 95% CI =1.11–1.75, *P*=0.0045).

**Figure 1:** Genotypes of the three *TIMD4-HAVCR1* SNPs and the risk of CHD and IS *P<0.017 was considered statistically significant (corresponding to *P*<0.05 after adjusting for three independent tests by the Bonferroni correction).

### Haplotypes and the risk of CHD and IS

As shown in the Figure 2, the haplotype of C-T-T (in order of the rs1501908, rs12522248, and rs2036402) was the commonest haplotype and represented ~60% of the sample. The haplotype of G-T-T was associated with an increased risk for CHD (adjusted OR =1.28, 95% CI =1.05–1.57, *P*=0.015), but the haplotype of G-C-T was associated with a decreased risk for CHD (adjusted OR =0.39, 95% CI =0.19–0.83, *P* =0.015). The haplotype of C-C-C was associated with an increased risk for IS (adjusted OR =1.35, 95% CI =1.02–1.80, *P* =0.037).

**Figure 2:** Haplotype frequencies of the three *TIMD4-HAVCR1* SNPs and the risk of CHD and IS The haplotypes consist of three alleles in order of the rs1501908, rs12522248, and rs2036402 SNPs; *P < 0.05.

### Genotypes and serum lipid levels

The association of the *TIMD4-HAVCR1* SNPs and serum lipid levels in controls is presented in Figure 3. Serum TG and LDL-C levels were different amongst the genotypes of the rs1501908 (*P*<0.01 for each), the rs1501908G allele carriers had lower TG and LDL-C levels than the rs1501908G allele noncarriers. Serum HDL-C levels were different amongst the genotypes of the rs12522248 (*P*<0.01), the rs12522248C allele carriers had lower HDL-C levels than the rs12522248C allele noncarriers.

**Figure 3:** Genotypes of the three *TIMD4-HAVCR1* SNPs and serum lipid levels in controls The value of TG was presented as median (interquartile range), and the difference amongst the genotypes was determined by the Kruskal–Wallis test. *P<0.017 was considered statistically significant (corresponding to *P*<0.05 after adjusting for three independent tests by the Bonferroni correction).

### Haplotypes and serum lipid levels

The association of the haplotypes and serum lipid levels is shown in Figure 4. The G-T-T haplotype carriers had higher LDL-C levels than the G-T-T haplotype noncarriers (*P*<0.01). The C-C-C haplotype carriers had lower HDL-C levels and higher TC/HDL-C ratio than the C-C-C haplotype noncarriers (*P*<0.01 for each).

**Figure 4:** Haplotypes of the three *TIMD4-HAVCR1* SNPs and serum lipid levels in controls The haplotypes consist of three alleles in the order of rs1501908, rs12522248, and rs2036402. The value of TG was presented as median (interquartile range), and the difference amongst the genotypes was determined by the Kruskal–Wallis test. *P<0.017 was considered statistically significant (corresponding to *P*<0.05 after adjusting for three independent tests by the Bonferroni correction). **A**: C-T-T; **B**: G-T-T; **C**: G-C-T; and **D**: C-C-C haplotypes.

### Interactions of the *TIMD4-HAVCR1* SNPs and drinking, smoking, BMI, age, and sex on serum lipid levels and the risk of CHD and IS

Table 3 shows the interactions of the *TIMD4-HAVCR1* SNPs and drinking, smoking, BMI, age, and sex on serum lipid levels and the risk of CHD and IS. The SNPs of rs1501908 and rs2036402 interacted with alcohol consumption to influence serum HDL-C levels (Figure 5A,B). The SNPs of rs1501908 and rs12522248 interacted with BMI ≥24 kg/m^2^ to modulate serum TC levels (Figure 5C,D). The rs12522248CT/CC genotypes interacted with BMI ≥24 kg/m^2^ to increase the risk of CHD (*P*<0.001). No interaction of the genotypes and smoking, age, and sex on the risk of CHD and IS was detected in our study populations.

**Figure 5:** Interactions of the *TIMD4-HAVCR1* SNPs and drinking, smoking, BMI, age, and sex on serum lipid levels The differences in serum HDL-C and TC levels amongst the genotypes were assessed using ANCOVA. The differences in serum TG levels amongst the genotypes were determined by the Kruskal–Wallis test. The interactions of the genotypes and alcohol consumption or BMI ≥24 kg/m^2^ on serum lipid levels were detected by using a factorial regression analysis after controlling for potential confounders (*P*_I_). Genotype and alcohol consumption or BMI ≥24 kg/m^2^ interaction increases serum lipid levels (↑). *P*_I_ ≤0.003 was considered statistically significant after Bonferroni correction (according to three SNPs and five interactive factors). **A**: rs1501908-drinking interaction on HDL-C; **B**: rs2036402-drinking interaction on HDL-C; **C**: rs1501908-BMI≥24 kg/m^2^ interaction on TC; and **D**: rs12522248-BMI≥24 kg/m^2^ interaction on TC.

**Table 3:** The *P*_I_ values for interactions of genotypes and drinking, smoking, and BMI on serum lipid levels and the risk of CHD and IS

SNP/factor	TC	TG	HDL-C	LDL-C	TC/HDL-C	ApoA1	ApoB	ApoA1/ApoB	CHD	IS
rs1501918										
Smoking	0.520	0.374	0.476	0.112	0.994	0.714	0.906	0.442	0.620	0.341
Drinking	0.268	0.246	<0.001	0.415	0.006	0.005	0.185	0.728	0.686	0.093
BMI	<0.001	0.005	0.290	0.004	0.005	0.706	0.046	0.054	0.556	0.923
Age	0.147	0.591	0.885	0.033	0.081	0.736	0.758	0.340	0.122	0.920
Sex	0.098	0.503	0.692	0.073	0.054	0.298	0.257	0.188	0.901	0.067
rs12522248										
Smoking	0.658	0.022	0.020	0.035	0.615	0.072	0.975	0.909	0.262	0.504
Drinking	0.700	0.618	0.134	0.383	0.007	0.404	0.639	0.355	0.183	0.864
BMI	0.001	0.010	0.037	0.083	0.013	0.135	0.207	0.066	<0.001	0.974
Age	0.869	0.459	0.288	0.497	0.077	0.628	0.308	0.016	0.072	0.681
Sex	0.131	0.811	0.142	0.069	0.049	0.016	0.011	0.431	0.842	0.502
rs2036402										
Smoking	0.709	0.492	0.441	0.081	0.678	0.097	0.507	0.253	0.743	0.371
Drinking	0.702	0.633	0.001	0.112	0.052	0.282	0.906	0.552	0.375	0.991
BMI	0.438	0.753	0.264	0.198	0.074	0.640	0.364	0.115	0.089	0.672
Age	0.653	0.782	0.066	0.348	0.423	0.666	0.209	0.059	0.565	0.587
Sex	0.354	0.851	0.445	0.195	0.186	0.029	0.032	0.792	0.693	0.814

*P*_I_≤0.003 was considered statistically significant after Bonferroni correction (according to three SNPs and five interactive factors).

### Interactions of the haplotypes and BMI on the risk of CHD

The interactions of several haplotypes and BMI ≥24 kg/m^2^ on the risk of CHD were also noted in the present study. As compared with the C-T-T haplotype in BMI <24 kg/m^2^, the haplotypes of C-T-T (OR =1.94, 95% CI =1.31–2.84), G-T-T (OR =2.33, 95% CI =1.63–3.33) and C-C-C (OR =2.56, 95% CI =1.54–4.28) in BMI ≥24 kg/m^2^ were associated with an increased risk of CHD. As compared with the same haplotype in BMI <24 kg/m^2^, the haplotypes of C-T-T (OR =1.94, 95% CI =1.31–2.87), G-T-T (OR =2.16, 95% CI =1.55–3.02) and C-C-C (OR =2.16, 95% CI =1.23–3.81) in BMI ≥24 kg/m^2^ were associated with an increased risk of CHD.

### Interactions of the haplotypes and BMI on the risk of IS

The interactions of several haplotypes and BMI ≥24 kg/m^2^ on the risk of IS were also observed in the present study. As compared with the C-T-T haplotype in BMI <24 kg/m^2^, the haplotypes of C-T-T (OR =1.64, 95% CI =1.11–2.41), G-T-T (OR =1.53, 95% CI =1.08–2.18), C-C-C (OR =2.27, 95% CI =1.39–3.69), and G-C-T (OR =2.62, 95% CI =1.09–6.32) in BMI ≥24 kg/m^2^ were associated with an increased risk of IS. As compared with the same haplotype in BMI <24 kg/m^2^, the haplotypes of C-C-T (OR =1.64, 95%CI =1.11–2.41), G-T-T (OR =1.66, 95% CI =1.18–2.33), and C-C-C (OR =1.98, 95% CI =1.16–3.88) in BMI ≥24 kg/m^2^ were associated with an increased risk of IS.

### Interactions of the *TIMD4-HAVCR1* SNPs and atorvastatin on serum lipid levels in hyperlipidemia

After 8-week treatment of atorvastatin, the levels of TC, TG, and LDL-C and the ratio of TC/HDL-C were significantly decreased in the hyperlipidemic patients (*P*<0.001 for all; Figure 6). There was no significant difference in serum HDL-C, ApoA1, and ApoB levels. We also found that the *TIMD4-HAVCR1* SNPs changed the effects of atorvastatin treatment on some serum lipid parameters. The rs1501908G and rs12522248C allele carriers had lower TC and LDL-C levels than the rs1501908G and rs12522248C allele noncarriers, respectively after atorvastatin treatment. The subjects with rs2036402TC genotype had lower TC and LDL-C levels than the subjects with rs2036402TT genotype after atorvastatin treatment. However, the subjects with rs1501908CC, rs12522248TT, and rs2036402TT genotypes had lower ApoA1 levels than the subjects with rs1501908CG/GG, rs12522248TC/CC, and rs2036402TC/CC genotypes, respectively after atorvastatin treatment (*P*<0.01 for all; Figure 6).

**Figure 6:** Effects of the *TIMD4-HAVCR1* SNPs on serum lipid levels at baseline and response to atorvastatin therapy in hyperlipidemia Genotype and atorvastatin interaction decreases serum lipid levels (↓); *P<0.001.

## Discussion

The present study showed that the genotypic and allelic frequencies of the rs12522248 SNP were different between controls and CHD or IS patients, and the rs12522248 genotypes or alleles were associated with the risk of CHD and IS in different genetic models. Strong LD was noted amongst these SNPs. The haplotype of C-T-T was the commonest haplotype. The G-T-T haplotype was associated with an increased risk for CHD, but the G-C-T haplotype was associated with a decreased risk for CHD. The C-C-C haplotype was associated with an increased risk for IS. The rs1501908G allele carriers had lower TG and LDL-C levels than the rs1501908G allele noncarriers. The rs12522248C allele carriers had lower serum HDL-C levels than the rs12522248C allele noncarriers. The G-T-T haplotype carriers had higher LDL-C levels than the G-T-T haplotype noncarriers. The C-C-C haplotype carriers had lower HDL-C levels and higher ratio of TC to HDL-C than the C-C-C haplotype noncarriers. The SNPs of rs1501908 and rs2036402 interacted with alcohol consumption to influence serum HDL-C levels. The SNPs of rs1501908 and rs12522248 interacted with BMI ≥24 kg/m^2^ to modify serum TC levels. The rs12522248TC/CC genotypes interacted with BMI ≥24 kg/m^2^ to increase the risk of CHD. The interactions of several haplotypes and some environment factors on the risk of CHD and IS were also observed.

Several previous studies have reported the association of many SNPs in the *TIMD4-HAVCR1* with one or more lipid traits [24,27–29]. However, not all researches have consistent findings. A previous GWAS showed that the rs1501908 SNP was associated with LDL-C in European ancestry, while a replication research conducted in Shanghai in China indicated that the rs1501908 variant in the *TIMD4-HAVCR1* was associated with TC, TG, LDL-C, and the ratio of TC to HDL-C [27]. Aguilar-Salinas et al. [29] showed that the rs2036402 SNP was associated with hypertriglyceridemia in Mexicans, but not in Caucasians. In the present study, we found that the rs1501908 SNP was associated with serum TG and LDL-C levels, which were partly consistent with the previous studies [24,27]. The rs12522248 SNP was associated with HDL-C levels, the 12522248C allele carriers had lower HDL-C concentrations than the 12522248C allele noncarriers, which was not reported previously. However, the association of the rs2036402 SNP and serum lipid profiles had not been detected. We also firstly showed that the G-T-T haplotype carriers had higher LDL-C levels than the G-T-T haplotype noncarriers; and the C-C-C haplotype carriers had lower HDL-C levels and higher TC/HDL-C ratio than the C-C-C haplotype noncarriers. The reasons for these diverse findings remain unclear. It may be owing to the impact of other uncertain variants and the different genetic background, lifestyle and diet in different ethnic groups. Another possible reason is that the sample size may not be enough to detect the exact association. Therefore, further investigations with larger sample size are needed to confirm our findings.

We also found that the genotypic and allelic frequencies of the *TIMD4-HAVCR1* rs12522248 SNP were different between controls and CHD or IS patients, the patients with CHD (19.0%) or IS (17.5%) had higher frequencies of rs12522248C allele than the controls (13.1%). The genotypes of the rs12522248 SNP were also associated with the risk of CHD and IS after the Bonferroni correction in different genetic models. The data in the International HapMap Project’s database have showed that the frequency of rs12522248C allele was 25.9% in European, 20.23% in Han Chinese in Beijing, 12.4% in Japanese, and 12.8% in Sub-Saharan African. As compared with the other populations, we found that the frequency of the rs12522248C allele in our study populations was lower than that in Han Chinese from Beijing, which might be caused by different sample sizes and Han Chinese from Beijing and Guangxi are different parts of Han. The prevalence of the rs12522248C allele was higher in European than in Chinese. These results suggest that the rs12522248C allele variation may have a racial/ethnic-specificity. *TIMD4*, present on macrophages and dendritic cells, plays a critical role in apoptotic cell clearance and regulates the number of phosphatidylserine-expressing activated T cells, whereas *HAVCR1* is expressed on activated T cells and is also found on dendritic cells and B cells [26]. Both apoptotic cell death and activated T cells play an important role in the maintenance of immune homeostasis in the atherosclerotic lesion [50–53]. A recent study showed that blockade of *TIMD4* aggravates atherosclerosis likely by prevention of phagocytosis of phosphatidylserine-expressing apoptotic cells and activated T cells by *TIMD4*-expressing cells, whereas *HAVCR1*-associated effects on atherosclerosis are related to changes in Th1/Th2 balance and reduced circulating regulatory T cells [26]. Another study detected that mice deficient for *TIMD4* or *HAVCR1* have increased susceptibility for autoimmunity, as shown by hyperactive T- and B-cell responses in *TIMD4*^−/−^ mice [54] and increased Th2 responses in *HAVCR1*^−/−^ mice [55]. In a human population-based study, Lind et al. [56] found an association between *HAVCR1* and plaque occurrence in carotid arteries using proteomic arrays. Zhao et al. [57] showed that *TIMD4* mRNA negatively correlated with LDL levels in mice having type II diabetes mellitus. In addition, the *TIMD4-HAVCR1* rs12522248 SNP in our present study was associated with serum HDL-C level, which has a strong effect on the risk of atherosclerosis related diseases. Taken together, the association of the rs12522248 SNP and the risk of CHD or IS might be owing to the immunosuppressive potency by regulating apoptotic cell clearance, the influence on adaptive immune responses, the association between the rs12522248 mutation and serum HDL-C levels or the influence of the other uncertain genes. To the best of our knowledge, this is the first report to evaluate the association between the rs12522248 SNP and the risk of CHD and IS. Therefore, these findings still need to be confirmed in the other populations with larger sample size.

The interactions of the *TIMD4-HAVCR1* SNPs and their haplotypes and some environmental factors on serum lipid levels and the risk of CHD and IS have not been reported previously. In the present study, we showed that two *TIMD4-HAVCR1* SNPs (rs1501918 and rs2036402) interacted with alcohol consumption to influence serum HDL-C levels. Two SNPs (rs1501918 and rs12522248) interacted with BMI ≥24 kg/m^2^ to modulate serum TC levels. The haplotypes of G-T-T and C-C-C interacted with smoking to increase the risk of CHD. The haplotypes of C-T-T, G-T-T, C-C-C, and G-C-T in BMI ≥24 kg/m^2^ were associated with an increased risk for CHD and IS. The rs12522248TC/CC genotypes interacted with BMI ≥24 kg/m^2^ to increase the risk of CHD. It is well known that heavy alcohol intake, smoking and obesity have an unfavourable effect on lipid profiles and atherosclerotic disease. Several case–control and cohort studies have described a J- or U-shaped association between alcohol intake and atherogenesis [58]. A moderate intake of alcohol when taken on a regular basis has been showed to protect against CHD death, which has been ascribed to the changes in serum HDL-C, TG and ApoA1 levels [59]. However, results from the Italian longitudinal study on aging also showed that alcohol consumption was associated with worse hematological values of TC and LDL-C levels [60]. A previous study reported that for every 1-kg decrease in body weight, TG decreased by 0.011 mmol/l and HDL-C increased by 0.011 mmol/l, which have beneficial effects on atherosclerotic disease. Another study about the correlation of BMI and atherogenic lipoprotein profile showed that overweight participants presented with 30% higher TG levels and 9% lower HDL-C concentration compared with normal-weight individuals. Therefore, the results of exposure to different environmental factors might further modify the effect of genetic variation on serum lipid levels and atherosclerotic disease in our study populations.

The interactions of the *TIMD4-HAVCR1* SNPs and statins are not well known. In the present study, we firstly showed that the *TIMD4-HAVCR1* SNPs changed the efficacy of atorvastatin on some serum lipid parameters. The rs1501908G and rs12522248C allele carriers had lower TC and LDL-C levels than the rs1501908G and rs12522248C allele noncarriers respectively after atorvastatin treatment. The subjects with rs2036402TC genotype had lower TC and LDL-C levels than the subjects with rs2036402TT genotype after atorvastatin treatment. However, the subjects with rs1501908CC, rs12522248TT, and rs2036402TT genotypes had lower ApoA1 levels than the subjects with rs1501908CG/GG, rs12522248TC/CC and rs2036402TC/CC genotypes respectively after atorvastatin treatment. These results suggest that the *TIMD4-HAVCR1* rs1501908G and rs12522248C allele carriers benefited more from atorvastatin therapy than the *TIMD4-HAVCR1* rs1501908G and rs12522248C allele noncarriers in decreasing serum TC and LDL-C levels. But the subjects with rs1501908CC, rs12522248TT, and rs2036402TT homozygotes might have a detrimental effect by decreasing serum ApoA1 levels after atorvastatin treatment.

## Study limitations

Although the present study provided interesting findings about the association of the *TIMD4-HAVCR1* SNPs and serum lipid phenotypes and the risk of CHD and IS, several potential limitations should be acknowledged in the present study. First, the sample size was relatively small compared with many GWASs and replication studies. Therefore, further studies with larger sample size are needed to confirm our results. Second, there were significant differences in the general characteristics between the control and patient groups. Although several confounders have been adjusted for the statistical analysis, we could not completely eliminate the potential effects of these factors on the results. Third, the association of the three SNPs and serum lipid levels in the CHD and IS groups was not analyzed because of the interference of lipid-lowering drugs. Finally, it is well known that both CHD and IS are the complex multifactorial diseases that are caused by genetic factors, various environmental factors and their interaction. Although we have detected the association of three SNPs and their haplotypes in the *TIMD4-HAVCR1* and the risk of CHD and IS, there are still many unmeasured environmental and genetic factors and their interactions, and this may result in some misinterpretation of our results.

## Conclusion

In the present study, we showed that the genotypic and allelic frequencies of the rs12522248 SNP were different between controls and patients, and the genotypes of the rs12522248 SNP were associated with the risk of CHD and IS in different genetic models. Several SNPs and their haplotypes in controls were associated with TG (rs1501918), LDL-C (rs1501918, G-T-T), HDL-C (rs12522248, C-C-C), and the ratio of TC to HDL-C (C-C-C). Several SNPs and their haplotypes interacted with alcohol consumption, smoking and BMI ≥24 kg/m^2^ to modify serum TC and HDL-C levels, and the risk of CHD and IS.

## Abbreviations

Apo: apolipoprotein
BMI: body mass index
CHD: coronary heart disease
GWAS: genome-wide association study
HAVCR1: hepatitis A virus cellular receptor 1
HDL-C: high-density lipoprotein cholesterol
IS: ischemic stroke
LD: linkage disequilibrium
LDL-C: low-density lipoprotein cholesterol
OR: odds ratio
SNP: single nucleotide polymorphism
TC: total cholesterol
TG: triglyceride
Th2: T-helper 2
TIMD4: T-cell immunoglobulin domain and mucin domain 4
TOAST: Trial of Org 10172 in Acute Stroke Treatment
95% CI: 95% confidence interval

## References

[1] MozaffarianD., BenjaminE.J., GoA.S., ArnettD.K., BlahaM.J., CushmanM. (2015) Heart disease and stroke statistics–2015 update: a report from the American Heart Association. Circulation 131, e29–322 10.1161/CIR.0000000000000152 25520374

[2] YamadaY., MatsuiK., TakeuchiI. and FujimakiT. (2015) Association of genetic variants with coronary artery disease and ischemic stroke in a longitudinal population-based genetic epidemiological study. Biomed. Rep. 3, 413–419 2613724710.3892/br.2015.440PMC4461855

[3] PasternakR.C., CriquiM.H., BenjaminE.J., FowkesF.G., IsselbacherE.M., McCulloughP.A. (2004) Atherosclerotic vascular disease conference: writing group I: epidemiology. Circulation 109, 2605–2612 10.1161/01.CIR.0000128518.26834.93 15173042

[4] YuX.H., FuY.C., ZhangD.W., YinK. and TangC.K. (2013) Foam cells in atherosclerosis. Clin. Chim. Acta 424, 245–252 10.1016/j.cca.2013.06.006 23782937

[5] StoneN.J., RobinsonJ.G., LichtensteinA.H., Bairey MerzC.N., BlumC.B., EckelR.H. (2014) 2013 ACC/AHA guideline on the treatment of blood cholesterol to reduce atherosclerotic cardiovascular risk in adults: a report of the American College of Cardiology/American Heart Association Task Force on Practice Guidelines. J. Am. Coll. Cardiol. 63, 2889–2934 10.1016/j.jacc.2013.11.002 24239923

[6] ChapmanM.J., GinsbergH.N., AmarencoP., AndreottiF., BorenJ., CatapanoA.L. (2011) Triglyceride-rich lipoproteins and high-density lipoprotein cholesterol in patients at high risk of cardiovascular disease: evidence and guidance for management. Eur. Heart J. 32, 1345–1361 10.1093/eurheartj/ehr112 21531743PMC3105250

[7] TsukinokiR., OkamuraT., WatanabeM., KokuboY., HigashiyamaA., NishimuraK. (2014) Blood pressure, low-density lipoprotein cholesterol, and incidences of coronary artery disease and ischemic stroke in Japanese: the Suita study. Am. J. Hypertens. 27, 1362–1369 10.1093/ajh/hpu059 24713850PMC4263939

[8] MeiL., FangX., MuL., LiuH., ZhangH., QinX. (2014) Association of serum high-density lipoprotein cholesterol level and risk of recurrent ischemic stroke. Zhonghua Xin Xue Guan Bing Za Zhi 42, 295–300 24924455

[9] ParkJ.H., HongK.S., LeeE.J., LeeJ. and KimD.E. (2011) High levels of apolipoprotein B/AI ratio are associated with intracranial atherosclerotic stenosis. Stroke 42, 3040–3046 10.1161/STROKEAHA.111.620104 21868729

[10] TeixeiraP.C., DucretA., FerberP., GaertnerH., HartleyO., PaganoS. (2014) Definition of human apolipoprotein A-I epitopes recognized by autoantibodies present in patients with cardiovascular diseases. J. Biol. Chem. 289, 28249–28259 10.1074/jbc.M114.589002 25170076PMC4192480

[11] LusisA.J., MarR. and PajukantaP. (2004) Genetics of atherosclerosis. Annu. Rev. Genomics Hum. Genet. 5, 189–218 10.1146/annurev.genom.5.061903.175930 15485348

[12] WillerC.J., SchmidtE.M., SenguptaS., PelosoG.M., GustafssonS., KanoniS. (2013) Discovery and refinement of loci associated with lipid levels. Nat. Genet. 45, 1274–1283 10.1038/ng.2797 24097068PMC3838666

[13] HataY. and NakajimaK. (2000) Life-style and serum lipids and lipoproteins. J. Atheroscler. Thromb. 7, 177–197 10.5551/jat1994.7.177 11521681

[14] BarnardR.J. (1991) Effects of life-style modification on serum lipids. Arch. Intern. Med. 151, 1389–1394 10.1001/archinte.1991.00400070141019 2064490

[15] NahrendorfM. and SwirskiF.K. (2015) Lifestyle effects on hematopoiesis and atherosclerosis. Circ. Res. 116, 884–894 10.1161/CIRCRESAHA.116.303550 25722442PMC4347940

[16] MatsuzawaY. (2001) Life style-related disease. Nihon Rinsho 59, 188–194 11197854

[17] OrdovasJ.M., RobertsonR. and CleirighE.N. (2011) Gene–gene and gene–environment interactions defining lipid-related traits. Curr. Opin. Lipidol. 22, 129–136 10.1097/MOL.0b013e32834477a9 21311326

[18] OrdovasJ.M. and ShenA.H. (2002) Genetics, the environment, and lipid abnormalities. Curr. Cardiol. Rep. 4, 508–513 10.1007/s11886-002-0115-4 12379174

[19] AndreassiM.G. (2009) Metabolic syndrome, diabetes and atherosclerosis: influence of gene–environment interaction. Mutat. Res. 667, 35–43 10.1016/j.mrfmmm.2008.10.018 19028510

[20] HellerD.A., de FaireU., PedersenN.L., DahlenG. and McClearnG.E. (1993) Genetic and environmental influences on serum lipid levels in twins. N. Engl. J. Med. 328, 1150–1156 10.1056/NEJM199304223281603 8455681

[21] IliadouA., LichtensteinP., de FaireU. and PedersenN.L. (2001) Variation in genetic and environmental influences in serum lipid and apolipoprotein levels across the lifespan in Swedish male and female twins. Am. J. Med. Genet. 102, 48–58 10.1002/1096-8628(20010722)102:1%3c48::AID-AJMG1388%3e3.0.CO;2-4 11471172

[22] MarenbergM.E., RischN., BerkmanL.F., FloderusB. and de FaireU. (1994) Genetic susceptibility to death from coronary heart disease in a study of twins. N. Engl. J. Med. 330, 1041–1046 10.1056/NEJM199404143301503 8127331

[23] TeslovichT.M., MusunuruK., SmithA.V., EdmondsonA.C., StylianouI.M., KosekiM. (2010) Biological, clinical and population relevance of 95 loci for blood lipids. Nature 466, 707–713 10.1038/nature09270 20686565PMC3039276

[24] KathiresanS., WillerC.J., PelosoG.M., DemissieS., MusunuruK., SchadtE.E. (2009) Common variants at 30 loci contribute to polygenic dyslipidemia. Nat. Genet. 41, 56–65 10.1038/ng.291 19060906PMC2881676

[25] FreemanG.J., CasasnovasJ.M., UmetsuD.T. and DeKruyffR.H. (2010) TIM genes: a family of cell surface phosphatidylserine receptors that regulate innate and adaptive immunity. Immunol. Rev. 235, 172–189 10.1111/j.0105-2896.2010.00903.x 20536563PMC2914464

[26] FoksA.C., EngelbertsenD., KuperwaserF., Alberts-GrillN., GonenA., WitztumJ.L. (2016) Blockade of Tim-1 and Tim-4 enhances atherosclerosis in low-density lipoprotein receptor-deficient mice. Arterioscler. Thromb. Vasc. Biol. 36, 456–465 10.1161/ATVBAHA.115.306860 26821944PMC4853762

[27] ZhangZ., TaoL., ChenZ., ZhouD., KanM., ZhangD. (2011) Association of genetic loci with blood lipids in the Chinese population. PLoS ONE 6, e27305 10.1371/journal.pone.0027305 22073310PMC3207848

[28] DoR., WillerC.J., SchmidtE.M., SenguptaS., GaoC., PelosoG.M. (2013) Common variants associated with plasma triglycerides and risk for coronary artery disease. Nat. Genet. 45, 1345–1352 10.1038/ng.2795 24097064PMC3904346

[29] Aguilar-SalinasC.A., Tusie-LunaT. and PajukantaP. (2014) Genetic and environmental determinants of the susceptibility of Amerindian derived populations for having hypertriglyceridemia. Metabolism 63, 887–894 10.1016/j.metabol.2014.03.012 24768220PMC4315146

[30] ChenQ., ReisS.E., KammererC.M., McNamaraD.M., HolubkovR., SharafB.L. (2003) Association between the severity of angiographic coronary artery disease and paraoxonase gene polymorphisms in the National Heart, Lung, and Blood Institute-sponsored Women's Ischemia Syndrome Evaluation (WISE) study. Am. J. Hum. Genet. 72, 13–22 10.1086/345312 12454802PMC378617

[31] XuY., WangW., ZhangL., QiL.P., LiL.Y., ChenL.F. (2011) A polymorphism in the ABCG1 promoter is functionally associated with coronary artery disease in a Chinese Han population. Atherosclerosis 219, 648–654 10.1016/j.atherosclerosis.2011.05.043 21722899

[32] AdamsH.P.Jr, BendixenB.H., KappelleL.J., BillerJ., LoveB.B., GordonD.L. (1993) Classification of subtype of acute ischemic stroke. Definitions for use in a multicenter clinical trial. TOAST. Trial of Org 10172 in Acute Stroke Treatment. Stroke 24, 35–41 10.1161/01.STR.24.1.35 7678184

[33] WuD.F., YinR.X., CaoX.L., ChenW.X., AungL.H., WangW. (2013) Scavenger receptor class B type 1 gene rs5888 single nucleotide polymorphism and the risk of coronary artery disease and ischemic stroke: a case–control study. Int. J. Med. Sci. 10, 1771–1777 10.7150/ijms.7044 24151447PMC3804801

[34] WuD.F., YinR.X., CaoX.L. and ChenW.X. (2014) Association between single nucleotide polymorphism rs1044925 and the risk of coronary artery disease and ischemic stroke. Int. J. Mol. Sci. 15, 3546–3559 10.3390/ijms15033546 24577316PMC3975353

[35] YangQ., YinR.X., ZhouY.J., CaoX.L., GuoT. and ChenW.X. (2015) Association of polymorphisms in the *MAFB* gene and the risk of coronary artery disease and ischemic stroke: a case–control study. Lipids Health Dis. 14, 79 10.1186/s12944-015-0078-2 26204962PMC4513700

[36] ZhouY.J., HongS.C., YangQ., YinR.X., CaoX.L. and ChenW.X. (2015) Association of variants in CELSR2-PSRC1-SORT1 with risk of serum lipid traits, coronary artery disease and ischemic stroke. Int. J. Clin. Exp. Pathol. 8, 9543–9551 26464717PMC4583949

[37] WangH., QiuQ., TanL.L., LiuT., DengX.Q., ChenY.M. (2009) Prevalence and determinants of diabetes and impaired fasting glucose among urban community-dwelling adults in Guangzhou, China. Diabetes Metab. 35, 378–384 10.1016/j.diabet.2009.03.006 19665414

[38] YangM., ChenP., JinH., XieX., GaoT., YangL. (2014) Circulating levels of irisin in middle-aged first-degree relatives of type 2 diabetes mellitus - correlation with pancreatic beta-cell function. Diabetol. Metab. Syndr. 6, 133 10.1186/1758-5996-6-133 25530809PMC4271516

[39] AungL.H., YinR.X., WuD.F., WangW., LiuC.W. and PanS.L. (2014) Association of the variants in the BUD13-ZNF259 genes and the risk of hyperlipidaemia. J. Cell. Mol. Med. 18, 1417–1428 10.1111/jcmm.12291 24780069PMC4124025

[40] LiaoP.J., XieR.B., YinR.X., WeiD.X., HuangJ., HuangF. (2015) Serum lipid profiles, the prevalence of dyslipidemia and the risk factors in two isolated Chinese minorities. Int. J. Clin. Exp. Med. 8, 19200–19211 26770556PMC4694456

[41] YinR.X., WuD.F., WuJ.Z., CaoX.L., AungL.H., MiaoL. (2012) Interactions of several lipid-related gene polymorphisms and cigarette smoking on blood pressure levels. Int. J. Biol. Sci. 8, 685–696 10.7150/ijbs.4401 22606049PMC3354626

[42] YinR.X., AungL.H., LongX.J., YanT.T., CaoX.L., HuangF. (2015) Interactions of several genetic polymorphisms and alcohol consumption on blood pressure levels. Biofactors 41, 339–351 10.1002/biof.1234 26354227

[43] ZhouB.F. (2002) Predictive values of body mass index and waist circumference for risk factors of certain related diseases in Chinese adults-study on optimal cut-off points of body mass index and waist circumference in Chinese adults. Biomed. Environ. Sci. 15, 83–96 12046553

[44] WildmanR.P., GuD., ReynoldsK., DuanX. and HeJ. (2004) Appropriate body mass index and waist circumference cutoffs for categorization of overweight and central adiposity among Chinese adults. Am. J. Clin. Nutr. 80, 1129–1136 1553165810.1093/ajcn/80.5.1129

[45] DenisJ.B. and VincourtP. (1982) Panorama des methodes statistiques d’analyse des interactions genotype X milieu. Agronomie 2, 219–230

[46] FinlayK.W. and WilkinsonG.N. (1963) The analysis of adaptation in a plant-breeding programme. Aust. J. Agric. Res. 14, 742–754 10.1071/AR9630742

[47] WoodJ.T. (1976) The use of environmental variables in the interpretation of genotype-environment interaction. Heredity 37, 1–7 10.1038/hdy.1976.61 1066339

[48] DenisJ.B. (1980) Analyse de regression factorielle. Biom. Praxim. 20, 1–34

[49] DenisJ.B. (1988) Two-way analysis using covariates 1. Statistics 19, 123–132 10.1080/02331888808802080

[50] TabasI. (2010) Macrophage death and defective inflammation resolution in atherosclerosis. Nat. Rev. Immunol. 10, 36–46 10.1038/nri2675 19960040PMC2854623

[51] KockxM.M., De MeyerG.R., MuhringJ., JacobW., BultH. and HermanA.G. (1998) Apoptosis and related proteins in different stages of human atherosclerotic plaques. Circulation 97, 2307–2315 10.1161/01.CIR.97.23.2307 9639374

[52] BuonoC., BinderC.J., StavrakisG., WitztumJ.L., GlimcherL.H. and LichtmanA.H. (2005) T-bet deficiency reduces atherosclerosis and alters plaque antigen-specific immune responses. Proc. Natl. Acad. Sci. U.S.A. 102, 1596–1601 10.1073/pnas.0409015102 15665085PMC547865

[53] WhitmanS.C., RavisankarP. and DaughertyA. (2002) IFN-gamma deficiency exerts gender-specific effects on atherogenesis in apolipoprotein E-/- mice. J. Interferon Cytokine Res. 22, 661–670 10.1089/10799900260100141 12162876

[54] CurtissM.L., GormanJ.V., BusingaT.R., TraverG., SinghM., MeyerholzD.K. (2012) Tim-1 regulates Th2 responses in an airway hypersensitivity model. Eur. J. Immunol. 42, 651–661 10.1002/eji.201141581 22144095PMC3528103

[55] Rodriguez-ManzanetR., SanjuanM.A., WuH.Y., QuintanaF.J., XiaoS., AndersonA.C. (2010) T- and B-cell hyperactivity and autoimmunity associated with niche-specific defects in apoptotic body clearance in TIM-4-deficient mice. Proc. Natl. Acad. Sci. U.S.A. 107, 8706–8711 10.1073/pnas.0910359107 20368430PMC2889349

[56] LindL., ArnlovJ., LindahlB., SiegbahnA., SundstromJ. and IngelssonE. (2015) Use of a proximity extension assay proteomics chip to discover new biomarkers for human atherosclerosis. Atherosclerosis 242, 205–210 10.1016/j.atherosclerosis.2015.07.023 26204497

[57] ZhaoP., WangH., LiT., LeiC., XuX., WangW. (2016) Increased T-cell immunoglobulin and mucin domain containing 4 (TIM-4) is negatively correlated with serum concentrations of interleukin-1beta in Type II diabetes. J. Diabetes 8, 199–205 10.1111/1753-0407.12276 25676395

[58] RimmE.B., WilliamsP., FosherK., CriquiM. and StampferM.J. (1999) Moderate alcohol intake and lower risk of coronary heart disease: meta-analysis of effects on lipids and hemostatic factors. Br. Med. J. 319, 1523–1528 10.1136/bmj.319.7224.1523 10591709PMC28294

[59] De OliveiraE.S.E.R., FosterD., McGee HarperM., SeidmanC.E., SmithJ.D., BreslowJ.L. (2000) Alcohol consumption raises HDL cholesterol levels by increasing the transport rate of apolipoproteins A-I and A-II. Circulation 102, 2347–2352 10.1161/01.CIR.102.19.2347 11067787

[60] PerissinottoE., BujaA., MaggiS., EnziG., ManzatoE., ScafatoE. (2010) Alcohol consumption and cardiovascular risk factors in older lifelong wine drinkers: the Italian longitudinal study on aging. Nutr. Metab. Cardiovasc. Dis. 20, 647–655 10.1016/j.numecd.2009.05.014 19695851

